The article "Three-Dimensional Reconstruction of Cerebrovascular and Algorithm Realization" was retracted in 2023. Reasons: signs of a paper mill; suspected computer-generated content; unreliable results or conclusions; lack of ethics approval or compliance.

# Three-Dimensional Reconstruction of Cerebrovascular and Algorithm Realization

**DOI:** 10.1155/2021/7422884

**Published:** 2021-11-24

**Authors:** Linfeng Li, Xiao-Jing Jia

**Affiliations:** Affiliated Hospital of Beihua University, Jilin 132011, China

## Abstract

**Objective:**

In the three-dimensional reconstruction of CT cerebrovascular medical image registration, a new optimization algorithm based on the relative position information between the contours of various blood vessels in the image is proposed.

**Methods:**

Using the rule that the center of gravity of the vascular tissue structure on the series of slices has continuity, find the registration relationship between the contours of the vessels in the two adjacent slices. Because the shape of cerebrovascular contour is relatively symmetrical, its center of gravity is slightly away from its geometric center. Therefore, the geometric center is used to replace the center of gravity, and the “mass” of each contour is calculated according to the area of each contour to achieve the registration of the blood vessel contour.

**Results:**

The method has the characteristics of global optimization and stronger robustness.

**Conclusion:**

The cerebrovascular image obtained by this method is more realistic and can be used for the import of various software, simulation training, and later research, which provides an effective method for preoperative simulation of cerebrovascular intervention surgery.

## 1. Introduction

The source image of three-dimensional reconstruction of CT cerebrovascular medical images is from the two-dimensional tomographic parallel scanning reconstruction image. An inevitable problem in the three-dimensional reconstruction process is the contour registration of blood vessel images. In recent years, people have conducted in-depth research on the technology of three-dimensional reconstruction of parallel medical two-dimensional tomography images and have achieved great development. Because the reconstructed three-dimensional object image is helpful for understanding and researching the anatomical structure of cerebral blood vessels, as well as the development of medical diagnosis and remote medical technology, it is generally believed that the computer-assisted 3D cerebrovascular automatic reconstruction technology mainly includes the following problems: (1) extracting the contour of the region of interest in the series of 2D tomographic reconstruction images; (2) finding the contour of each contour between adjacent faults quasirelationship, that is, to determine which contours belong to the same cerebrovascular anatomy; (3) using these registration relationships to reconstruct the contour of the cerebrovascular anatomy tissue of interest from the series of two-dimensional tomographic reconstruction image contours; (4) the reconstructed cerebral blood vessels are displayed with a three-dimensional effect.

The article "Three-Dimensional Reconstruction of Cerebrovascular and Algorithm Realization" was retracted in 2023. Reasons: signs of a paper mill; suspected computer-generated content; unreliable results or conclusions; lack of ethics approval or compliance.

As we all know, the contour information in the image is extracted mainly by calculating the gray value “gradient” at each pixel point, that is, the place where the gradient value is large is usually the location of the contour, and a series of template operators have been developed on this idea. The designed template based on directional partial derivative integration has better effect. In terms of contour registration, the method proposed in [1] is to project the contour center to adjacent faults. If a contour center on adjacent faults falls within a certain threshold distance from the projection point, it is considered that the two contours are registered. However, considering the process of scanning and reconstruction, the relative position of two-dimensional fault images may be shifted, and this method only depends on the local position of the contour for registration in isolation; it is likely to produce large errors. Therefore, this method can only reach the local optimum, not the global optimum. In addition, due to the different size of the contours, the above threshold is not single, so it is not easy to determine.

A new method proposed in this paper is based on the internal information of the cerebral blood vessels (information of the mutual positions between the contours) based on the two-dimensional tomographic image, that is, the use of the cerebral vascular anatomy to have the continuity of the center of gravity on the series of slices regularly find the registration relationship between contours in two adjacent two-dimensional tomographic images. This method has the characteristics of global optimality and strong robustness [2].

## 2. Materials and Methods

After a series of image processing, the original medical image can extract the outline of cerebrovascular tissue on each two-dimensional tomographic image, as shown in Figure 1.

There are several vascular tissue contours on the same two-dimensional tomographic image, which can be represented by *Q*(*z*)={*Ct*_*i*_, *i*=0,1,2,…, *N*_*s*−1_}, where *Q*(*z*) represents the two-dimensional tomographic image with cylindrical coordinate *z*, and *N*_*s*_ is the number of contours on the tomographic image. By calculating the center of gravity *C*_*i*_=(*x*_*i*_, *y*_*i*_, *z*_*i*_) of each cerebrovascular contour *Ct*_*i*_, the set of center of gravity points *C*(*z*)={*C*_*i*_, *i*=0,1,2,…, *N*_*s*−1_} can be obtained, as shown in Figure 2.

However, in actual calculations, considering that the shape of the cerebrovascular contour is relatively symmetrical, its center of gravity is slightly away from its geometric center. Therefore, the geometric center can be used to replace the center of gravity, and then the “mass” can be obtained according to the area of each contour. Practice has proved that this replacement can greatly reduce the computational complexity. When the mass density of the objects represented by each contour in the two-dimensional tomography image is the same, the “quality” of each contour is proportional to the area it surrounds (using prior knowledge, different contours and weights can be given according to the actual situation to reflect the difference of density). In CT two-dimensional medical tomography of cerebrovascular, the contour of vascular tissue on the section is almost circular. In order to reduce the calculation complexity, this article will perform the following calculation: define the radius of the contour *Ct*_*i*_ as *r*_*i*_=*γ*_*i*_/2*π*, and *p*_*i*_ is the perimeter of contour *Ct*_*i*_. Since the mass of *Ct*_*i*_ is proportional to the area enclosed by the contour, that is, proportional to the square of the radius, its mass *m*_*i*_ can be expressed as

(1) $$\begin{array}{c} m_{i}=\gamma_{i}^{2}\pi \lambda_{i}. \end{array}$$

Among them, *λ*_*i*_ is the density of the contour *Ct*_*i*_. For the contour with the inner contour, the quality should also subtract the part included in the inner contour, namely,

(2) $$\begin{array}{c} m_{i}=\pi \lambda_{i}\left(r_{i}^{2}-\underset{i\in CI\left(i\right)}{\sum }r_{i}^{2}\right). \end{array}$$

Among them, *CI*(*i*) is the set of inner contours contained in the contour *Ct*_*i*_. When the mass density of the objects represented by each contour is the same, *πλ*_*i*_=1,  *i*=1,2,3,…, *N*_*s*_ is taken for convenience of calculation. After finding the center of gravity and “mass” of each contour in the 2D tomographic image, the common gravity center position *Cg*(*z*) of the 2D tomographic image can be calculated. The center of gravity is shown in Figure 2.

(3) $$\begin{array}{c} Cg\left(z\right)=\left(\frac{\sum_{i}^{N_{s-1}}m_{i}x_{i}}{\sum_{i}^{N_{s-1}}m_{i}},\frac{\sum_{i}^{N_{s-1}}m_{i}y_{i}}{\sum_{i}^{N_{s-1}}m_{i}}\right)z. \end{array}$$

Let *C*^*u*^={*C*_*i*_^*u*^, *i*=0,1,2,…, *N*_*u*−1_} represent the center of gravity of each contour of the upper 2D tomographic image, where *C*_*i*_^*u*^=(*x*_*i*_^*u*^, *y*_*i*_^*u*^, *z*_*i*_^*u*^), the common center of gravity of the upper 2D tomographic image is *C*_*g*_^*u*^, and *C*^*l*^={*C*_*i*_^*l*^, *i*=1,2,3,…, *N*_*l*−1_} represents the center of gravity of each contour of the lower 2D tomographic image, where *C*_*i*_^*l*^=(*x*_*i*_^*l*^, *y*_*i*_^*l*^, *z*_*i*_^*l*^), the lower 2D tomographic image. The common center of gravity of the scanned image is *C*_*g*_^*u*^. *N*_*u*_ and *N*_*l*_ are the numbers of layer contours of the upper and lower two-dimensional tomography images, respectively. In this paper, we take the two-dimensional tomographic image with a large number of contours to the two-dimensional tomographic image with a small number to find the contour registration relationship, so we might as well set *N*_*u*_≻*N*_*l*_; otherwise, we just need to reverse the order of the upper and lower faults in the following description of the method. The contour registration algorithm is as follows:

(1) For each contour *Ct*_*i*_^*u*^ of the upper fault, the (*x*, *y*) coordinate (*x*_*i*_^*u*^, *y*_*i*_^*u*^) of its center of gravity is converted into a polar coordinate (*p*_*i*_^*u*^, *ϕ*_*i*_^*u*^) relative to the common center of gravity *C*_*g*_^*u*^. Similarly, for each contour *Ct*_*j*_^*l*^ of the lower fault, its center of gravity (*x*, *y*). The coordinate (*x*_*i*_^*l*^, *y*_*i*_^*l*^) is transformed into the polar coordinate (*p*_*i*_^*l*^, *ϕ*_*i*_^*l*^) relative to the common center of gravity *C*_*g*_^*l*^ so that for the polar coordinate (*p*_*i*_^*l*^, *ϕ*_*i*_^*l*^) of the center of gravity of each contour of the upper fault, there must be a contour *Ct*_*j*_^*l*^ in the lower fault, if the polar coordinate (*p*_*i*_^*l*^, *ϕ*_*i*_^*l*^) of the center of gravity of the contour is closest to it, and the contour size is also the most similar, then this pair of contours is considered to be a registered contour.
In addition, when determining the contour registration relationship, the following three factors should be considered: (1) the radius value of their center of gravity polar coordinates is the closest; (2) the angle of their center of gravity polar coordinates is the closest; (3) their outline shape and the size are the most similar.
This is because there is obviously no registration relationship between contours that differ greatly in amplitude (as shown in Figure 3(a), contour will obviously not register with contour *C* in Figure 3(b)), so in the calculation, it is only necessary to find the registration relationship between the contours whose amplitudes are different within a certain threshold on the adjacent two-dimensional tomographic images. Set in the contour of the lower fault, and the difference between the center of gravity of the upper fault contour *Ct*_*i*_^*u*^ and the polar coordinate amplitude within the threshold value *θ* is *PM*_*i*_={*C*_*i*1_^*tl*^, *C*_*i*2_^*tl*^ … *C*_*iN*_^*tl*^} (such as the contour A in Figure 3(a)), this set corresponds to the fan in Figure 3(b) (A collection of outlines within the area).
(2) Make a measurement function *f*(*i*, *j*) to measure the possibility of registration of each contour in the contours *Ct*_*i*_^*u*^ and *PM*_*i*_:
  (4) $$\begin{array}{c} f\left(i,j\right)=\left|p_{i}^{u},p_{j}^{l}\right|+\alpha \left|\phi_{i}^{u},\phi_{j}^{l}\right|+\beta \left|r_{i}^{u},r_{j}^{l}\right|. \end{array}$$

Among them, *α* and *β* are the adjustment factors to adjust these three proportions, the specific value can be determined by experiment (in the following, given by the experiment). The three subitems in equation (4) correspond to the above three factors to be considered, of which the first item is used to measure the difference in polar coordinate radius values; the second item is used to measure the difference in polar coordinate amplitude angles. Three items are used to measure the similarity of the outline size.

The article "Three-Dimensional Reconstruction of Cerebrovascular and Algorithm Realization" was retracted in 2023. Reasons: signs of a paper mill; suspected computer-generated content; unreliable results or conclusions; lack of ethics approval or compliance.

Here, there is a situation that needs to be noted that because the common center of gravity of the two-dimensional tomographic image will move to a certain extent in adjacent faults, the change in the angle of the adjacent faults will be greater for the contours closer to the common center of gravity In this way, the abovementioned method of registering only contours with small distances between angles is not applicable. The solution is to set a threshold Ψ, and then, for contour lines, the distance between the center of gravity and the common center of gravity is greater than Ψ contour lines, using the above method. Conversely, for a contour whose distance between the center of gravity of the contour and the common center of gravity is less than Ψ, compare the value of the metric function *f* (*I, j*) with all contours of the lower fault to find the optimal registration contour. In this way, the registration relationship of each contour between adjacent two-dimensional tomographic images is determined. The obvious advantage of this method is that it has good globality, which makes full use of the relative between the contours in the same two-dimensional tomographic image. And the calculation is simple and fast and has good real-time.

## 3. Result

In order to test the effect of the registration algorithm in this paper, a method is designed to test the above registration algorithm. That is, first, *N* points are randomly generated on the coordinate plane with uniform probability as the center of gravity of the contour, and then *N* random samples of the normal distribution with mean *μ*_*r*_ and variance *σ*_*r*_ are generated. The sampling value of the state distribution is the radius, and a circle is used to represent a contour. In this way, the radius of most contours is near the mean *μ*_*r*_, and only a few circles have a larger or smaller radius, which is consistent with the actual situation. In this way, a two-dimensional tomographic image is constructed. Then, the following method is used to construct its adjacent two-dimensional tomographic image, with its coordinates offset by an average value of 0 and a random sampling value of the normal distribution with a variance of *σ*_*xy*_, that is, to move the center of the circle on the adjacent fault to a smaller position. To simulate the situation where the cerebrovascular tissue is displaced on adjacent faults, for each radius value of the circle, add a random sample of normal distribution with mean value 0 and variance *σ*_*r*_ to simulate cerebrovascular disease, the case where the tissue shape becomes thicker and thinner. Then, use each new center and radius value as a circle to generate a contour that is registered with the previous image so that a new adjacent 2D tomographic image is obtained [3].

The article "Three-Dimensional Reconstruction of Cerebrovascular and Algorithm Realization" was retracted in 2023. Reasons: signs of a paper mill; suspected computer-generated content; unreliable results or conclusions; lack of ethics approval or compliance.

Since the adjacent two-dimensional tomographic images are constructed using the above method, each contour registration relationship is known, as long as the above contour registration algorithm is used to find the registration relationship, and then the results obtained with the contour of the known registration relationship comparison can verify the correctness and pros and cons of the algorithm. The ratio of the number of contours correctly defined to the total number of contours defined here is the registration accuracy. Let the length and width of the two-dimensional tomography image be 512 each and the mean value *μ*_*r*_ of the radius of the contour be a reference. The registration accuracy rate is the average of 200 calculations. In this paper, several different parameters are selected for testing, and the following results are obtained. Figure 3 is the relationship between the registration accuracy of contours with different average radius *μ*_*r*_ and the number of contours *N* [4].

It can be seen from Figure 3 (1) the registration accuracy rate is mostly 0.93∼1; when the average radius of the contour is small, it can reach more than 0.96. This shows that the accuracy of the algorithm in this paper is very high; (2) the registration accuracy rate has a tendency to decrease with the increase in the number of contours in the same two-dimensional tomographic image, because the number of contours increase., The contour becomes “crowded,” and the ambiguous registration situation also increases accordingly; (3) when the average radius of the contour becomes larger and other parameters remain unchanged, the registration accuracy rate decreases, which is also because of the two-dimensional tomographic image. The outline inside becomes crowded [5].

The article "Three-Dimensional Reconstruction of Cerebrovascular and Algorithm Realization" was retracted in 2023. Reasons: signs of a paper mill; suspected computer-generated content; unreliable results or conclusions; lack of ethics approval or compliance.

It can be clearly seen from Figure 4 that the greater the *σxy*/*μr* and *σ′r*/*μr*, that is, the greater the change in the position of the contour and the radius of the contour between adjacent faults, the smaller the registration accuracy. This corresponds to the actual situation, that is, the larger the distance between adjacent two-dimensional scanned images, the greater the positional offset and the corresponding reduction in similarity, which will inevitably cause registration errors. Figure 4 shows that the change of contour size has a greater impact on the registration accuracy [6].

It can be seen from Figure 5 that when determining the size of *α* in equation (4), it can be calculated according to the different average radius of the profile. As *α* increases, the registration accuracy rate increases quickly, but after *α* reaches a certain level, the registration accuracy rate no longer increases significantly. According to Figure 5, this paper takes *α* at 20～25 as its ideal value.

It can be seen from Figure 6 that when determining the size of *β* in equation (4), it is found that when *β* is smaller, the registration accuracy rate is the largest; if *β* is increased again, the accuracy rate will be significantly reduced. According to Figure 6, the ideal value of *β* is 4–6.

## 4. Discussion

### 4.1. Image Input

Three consecutive 512 × 512 cerebrovascular medical tomography images were extracted from the 212 images. The thickness of the tomography was 1 mm, which was used as the algorithm experimental analysis object. Among them, Figure 7 is a scanned image of a noninvasive cerebral blood vessel after adding a contrast agent.  Figure 8 is an image of an ischemic cerebral blood vessel obtained by an edge extraction algorithm [7].

### 4.2. Algorithm Experiment

Comparative analysis of results: since the graphic registration method proposed in [8] has local optimal characteristics, the graphic registration method proposed in [8] is basically similar to the method proposed in this paper in a certain local reconstruction. Methods: the three-dimensional reconstruction of the image shows some interference, which can no longer fully meet the clinical application. From the perspective of the effect of reconstructed images, the method proposed in this paper is superior to the former, overcomes the above advantages, and basically satisfies the clinical application.  Figure 9 shows the reconstruction of three-dimensional images using the algorithm proposed in this paper.

The article "Three-Dimensional Reconstruction of Cerebrovascular and Algorithm Realization" was retracted in 2023. Reasons: signs of a paper mill; suspected computer-generated content; unreliable results or conclusions; lack of ethics approval or compliance.

## 5. Conclusion

Aiming at the common problem encountered in the process of three-dimensional reconstruction of cerebral blood vessels in CT cerebrovascular medical tomography images, the problem of blood vessel contour registration, a new algorithm based on the relative position information between each contour of the cerebral vascular anatomy in the image is proposed. That is to use the continuity of the position of the center of gravity of the cerebral vascular anatomy on a series of cross-sections to find the registration relationship between the contours in two adjacent faults. At the same time, a general method is designed and the algorithm is tested. The result proves that the effect of this method is obvious.

## Figures and Tables

**Figure 1:** Extraction of cerebrovascular tissue contours on the tomograms of adjacent scan images.

**Figure 2:** Tissue contour on the same scan image.

**Figure 3:** The relationship between the accuracy and the number of contours *N*.

**Figure 4:** The relationship between the accuracy and *σxy*/*μr*, *σ′r*/*μr*.

**Figure 5:** Experiment to determine the value of *α*.

**Figure 6:** Experiment to determine the value of *β*.

**Figure 7:** The cerebral vascular scan image with contrast agent.

**Figure 8:** Cerebrovascular edge extraction.

**Figure 9:** Reconstruction of three-dimensional images using the algorithm proposed in this paper.

## Data Availability

The data used to support the findings of this study are available from the corresponding author upon request.
